# Caspase-1 regulates Ang II-induced cardiomyocyte hypertrophy via up-regulation of IL-1β

**DOI:** 10.1042/BSR20171438

**Published:** 2018-03-16

**Authors:** Yunlong Bai, Xi Sun, Qun Chu, Anqi Li, Ying Qin, Yanyao Li, Er Yue, Hui Wang, GuiYang Li, Syeda Madiha Zahra, Chaorun Dong, Yanan Jiang

**Affiliations:** 1 Department of Pharmacology (State-Province Key Laboratories of Biomedicine- Pharmaceutics of China, Key Laboratory of Cardiovascular Medicine Research, Ministry of Education), College of Pharmacy, Harbin Medical University, Harbin 150081, P.R. China; 2 Chronic Disease Research Institute, Translational Medicine Research and Cooperation Center of Northern China, Heilongjiang Academy of Medical Sciences, Harbin 150081, P.R. China

**Keywords:** Cardiac hypertrophy, caspase-1, IL-1β, pyroptosis

## Abstract

Cardiac hypertrophy is a compensatory response to stress or stimuli, which results in arrhythmia and heart failure. Although multiple molecular mechanisms have been identified, cardiac hypertrophy is still difficult to treat. Pyroptosis is a caspase-1-dependent pro-inflammatory programmed cell death. Caspase-1 is involved in various types of diseases, including hepatic injury, cancers, and diabetes-related complications. However, the exact role of caspase-1 in cardiac hypertrophy is yet to be discovered. The present study aimed to explore the possible role of caspase-1 in pathogenesis of cardiac hypertrophy. We established cardiac hypertrophy models both *in vivo* and *in vitro* to detect the expression of caspase-1 and interleukin-1β (IL-1β). The results showed that caspase-1 and IL-1β expression levels were significantly up-regulated during cardiac hypertrophy. Subsequently, caspase-1 inhibitor was co-administered with angiotensin II (Ang II) in cardiomyocytes to observe whether it could attenuate cardiac hypertrophy. Results showed that caspase-1 attenuated the pro-hypertrophic effect of Ang II, which was related to the down-regulation of caspase-1 and IL-1β. In conclusion, our results provide a novel evidence that caspase-1 mediated pyroptosis is involved in cardiac hypertrophy, and the inhibition of caspase-1 will offer a therapeutic potential against cardiac hypertrophy.

## Introduction

Cardiac hypertrophy is a common response of heart to a variety of stimuli, which could be divided into physiological hypertrophy and pathological hypertrophy [1,2]. Pathological hypertrophy, is a major change of heart disease and considered as a critical risk factor of heart failure and is often associated with arrhythmia [3,4]. The cardiac dysfunction reflects the distinct pathogenesis of pathological cardiac hypertrophy. Although many pathways and targets have been reported to be effective, pathological cardiac hypertrophy inevitably leads to the unfavorable outcomes of heart failure [5,6]. Therefore, it is important to find novel therapeutic targets for hypertrophy.

Pyroptosis is a kind of caspase-1 or caspase-11-dependent programmed cell death [7,8]. Different from other programmed cell deaths, pyroptosis is a consequence of caspase-1 or caspase-11 activation in inflammasomes [9–12]. During pyroptosis, the activation of caspase-1 could cleave pro-interleukin-1β (IL-1β) to bioactive IL-1β [13]. Studies have demonstrated that pyroptosis is involved in various types of diseases, including hepatic injury, cancers, and diabetes-related complications [14–16]. For cancer cells, loss of caspase-1 gene expression was observed in human prostate cancer and human hepatocellular carcinoma. The activation of pyroptosis may promote cell death and thus exert anticancer properties [15,17]. Although the importance of pyroptosis was identified in different kinds of diseases, little was known about the role of pyroptosis in cardiac hypertrophy.

To our knowledge, this is the first study to demonstrate that caspase-1-mediated pyroptosis plays a role in the pathogenesis of the cardiac hypertrophy and caspase-1 inhibitor AC-YVAD-CMK can mitigate cardiac hypertrophy induced by angiotensin II (Ang II).

## Materials and methods

### Ethics statement

The study was approved by the ethics committee of Harbin Medical University, and all experimental procedures were approved by the Animal Care and Use Committee of Harbin Medical University. Our study was performed in accordance with the recommendations of the Guide for the Care and Use of Laboratory Animals, published by the US National Institutes of Health (NIH Publication number 85-23, revised 1996).

### Mice model of pressure overload-induced cardiac hypertrophy

Pressure overload was imposed on the heart of mice by transverse aortic constriction (TAC). Adult mice (6-8 weeks) were anesthetized and placed in supine position and a midline cervical incision was made to expose the trachea. Then, the chest of mouse was opened and thoracic aorta was identified. A 5-0 silk suture was placed around the transverse aorta and tied around a 26-gauge blunt needle, which was subsequently removed. The chest was closed and the animals were kept ventilated until recovery of autonomic breath. Twenty-four mice were randomly divided into Sham and TAC groups. After treatment, the cardiac tissues were obtained for the following detection.

### Primary culture of neonatal mouse cardiomyocytes

Neonatal mouse cardiomyocytes were isolated from 1 to 3 days old C57BL/6 mouse hearts. Briefly, hearts were rapidly removed from neonatal mice and washed to remove blood and debris. Whole hearts were then cut into small pieces and dissociated into single cells by digestion with trypsin, EDTA solution (Solarbio, Beijing, China). The suspension was collected and added to Dulbecco’s modified Eagle’s medium (DMEM) nutrient mixture (HyClone, Logan, UT, U.S.A.) containing 10% FBS (BI, Kibbutz Beit Haemek, Israel) to end digestion. The above steps were repeated until all the tissues were digested. The collected cell suspension was filtered and centrifuged at 1500 rpm for 5 min to obtain cells. After centrifugation, cells were suspended in DMEM (HyClone, Logan, UT, U.S.A.) with 10% FBS, and precultured in humidified incubator (95% air, 5% CO_2_) for 1.5 h to obtain cardiac fibroblasts for their selective adhesion. Then, the suspended cardiomyocytes were plated in another dish. Culture medium was renewed after 48 h.

### Ang II-induced cardiomyocyte hypertrophy *in vitro*

Ang II treatment was used to induce cardiomyocyte hypertrophy. In our experiments, cardiomyocytes were incubated with 100 nmol/l Ang II for 48 h. The serum-free medium containing Ang II was changed every 24 h. Cardiomyocytes were prepared for immunofluorescence staining, real-time PCR, and Western blot assays. For immunofluorescence staining, monoclonal antibody against sarcomeric α-actinin (Sigma, St. Louis, Missouri, U.S.A.) was added at dilutions of 1:200. Nuclear staining was performed with Hoechst (Sigma, St. Louis, Missouri, U.S.A.). Immunofluorescence was examined under a fluorescence microscope (Zeiss, Heidenheim, Baden-Wuerttemberg, Germany). The surface areas of individual cardiomyocytes were measured using Image-Pro Plus software, which was normalized to control group. To avoid human error, at least five independent zones were selected in one slide and the quantitation was performed blinded by two individuals.

### Real-time PCR

The total RNA samples were extracted from cardiomyocytes or cardiac tissues using the TRIzol reagent (TaKaRa, Otsu, Shiga, Japan). Total RNA for 500 ng was reverse transcribed to cDNA using Reverse Transcriptase Master Kit (Toyobo, Osaka, Japan) according to the manufacturer’s instructions. Real-time PCR was performed on ABI 7500 fast system (Applied Biosystems, Carlsbad, CA, U.S.A.) using SYBR Green I (Toyobo, Osaka, Japan). GAPDH served as an internal control. The relative quantitation of gene expression was determined using the 2^−ΔΔCT^ method.

### Western blot

Total protein was extracted from cardiomyocytes or cardiac tissues. The suspension was subjected to 10% acrylamide gel electrophoresis (SDS/PAGE) followed by electrotransfer onto PVDF membranes (Roche Applied Science, Pleasanton, CA, U.S.A.). After blocking with 5% (w/v) BSA dissolved in TBST solution (10 mM Tris-HCl adjusted to pH 7.4 with HCl, 150 mM NaCl, 0.05% (v/v) Tween 20) for 2 h, the membranes were incubated at 4°C overnight with primary antibodies of caspase-1 (Cell Signaling, Danvers, Massachusetts, U.S.A.), IL-1β and GAPDH (ZSGB-BIO, Beijing, China), followed by incubation with horserasish peroxidase (HRP)-labeled goat anti-mouse IgG or anti-rabbit IgG (1:1000) (ZSGB-BIO, Beijing, China) for 1 h. Western blot bands were quantitated using Quantity One software. GAPDH served as an internal control.

### Hematoxylin and Eosin staining

Cardiac tissues were fixed in 4% paraformaldehyde followed by dehydration. The processed samples were embedded in paraffin and cut into 5-μm thick sections using tissue-processing equipment. The sections were deparaffinized and stained with Hematoxylin and Eosin (HE) for histological analysis.

### Immunohistochemistry

Cardiac tissues were fixed with 4% buffered paraformaldehyde, dehydrated, and embedded in paraffin. Five-micrometer thick sections were deparaffinized, rehydrated, and rinsed in distilled water. Antigen unmasking was carried out by water vapor heating in citrate buffer for 20 min. All sections were immunostained with the primary antibody against caspase-1 and IL-1β at 4°C overnight. After incubation with the secondary antibody, the sections were stained with diaminobenzidine.

### Statistical analysis

All the experiments were repeated five times, and the results were from one representative experiment. Data are expressed as mean ± S.E.M. and were analyzed with SPSS 13.0 software. Statistical comparisons between two groups were performed using Student’s *t*test. Statistical comparisons amongst multiple groups were performed using ANOVA, followed by Bonferroni’s post hoc test. A two-tailed *P*<0.05 was considered statistically significant. Graphs were generated using GraphPad Prism 5.0.

## Results

### Cleaved caspase-1 and IL-1β expression levels were up-regulated in myocardium of mice in response to acute pressure overload

The results of HE staining showed that TAC induces cardiac hypertrophy in mice (Figure 1A). High expression of cleaved caspase-1 was observed in the TAC group compared with sham group. Consistently, the downstream factor that cleaved IL-1β was also up-regulated in the myocardium of TAC-operated mice (Figure 1B). Real-time PCR assay showed that *capsase-1* and *IL-1β* mRNA expression levels were up-regulated in TAC group compared with control group (Figure 1C,D). Correspondingly, Western blot assay further confirmed the high protein expression levels of cleaved caspase-1 and its downstream factors cleaved IL-1β protein in TAC group compared with control group (Figure 1E,F). These results verified that the activation of pyroptosis is associated with cardiac hypertrophy.

**Figure 1:** The cleaved caspase-1 and IL-1β expression were up-regulated in myocardium from TAC mice model (**A**) The histopathological changes in Sham and TAC groups. (**B**) The immunohistochemical staining of cleaved caspase-1 and IL-1β in Sham and TAC groups. (**C**,**D**) *Caspase-1* and *IL-1β* mRNA expression levels were up-regulated in myocardium form TAC operated mice. (**E**,**F**). Cleaved caspase-1 and IL-1β protein expression levels were up-regulated in myocardium form TAC operated mice. GAPDH served as the internal control. *P<0.05 compared with Sham, ***P<0.001 compared with Sham; *n*=5.

### Ang II up-regulates cleaved caspase-1 and IL-1β expression in cardiomyocytes

We further examined the expression of cleaved caspase-1 and IL-1β in Ang II-treated cardiomyocytes. Neonatal mouse cardiomyocytes were exposed to Ang II (100 nmol/l) for 48 h. The *caspase-1* and *IL-1β* mRNA expression levels were up-regulated in Ang II-treated cardiomyocytes (Figure 2A,B). Consistently, the cleaved caspase-1 and IL-1β protein expression levels were also up-regulated in Ang II-treated cardiomyocytes (Figure 2C,D).

**Figure 2:** Ang II up-regulates cleaved caspase-1 and IL-1β expression in cardiomyocytes (**A**,**B**) *Caspase-1* and *IL-1β* mRNA expression levels were up-regulated in cardiomyocytes treated with Ang II. (**C**,**D**) Cleaved caspase-1 and IL-β protein expression levels were up-regulated in cardiomyocytes treated with Ang II. GAPDH served as the internal control. *P<0.05 compared with Control, **P<0.01 compared with Control; *n*=3.

### Caspase-1 inhibitor down-regulates cleaved caspase-1 and IL-1β expression in Ang II-treated cardiomyocytes

To further understand the correlation of pyroptosis and cardiac hypertrophy, caspase-1 inhibitor was used to detect the role of cleaved caspase-1 in cardiac hypertrophy. Cardiomyocytes were treated with vehicle, Ang II, and Ang II + AC-YVAD-CMK, respectively. The up-regulation of cleaved caspase-1 and IL-1β induced by Ang II was reversed by co-treatment with AC-YVAD-CMK in cardiomyocytes (Figure 3A–D).

**Figure 3:** Caspase-1 inhibitor down-regulates cleaved caspase-1 and IL-1β expression in Ang II treated cardiomyocytes (**A**,**B**) Caspase-1 inhibitor down-regulates *caspase-1* and *IL-1β* mRNA expression levels in Ang II-treated cardiomyocytes. (**C**,**D**) Caspase-1 inhibitor down-regulates caspase-1 and IL-1β protein expression levels in Ang II-treated cardiomyocytes. GAPDH served as the internal control. **P<0.01 compared with Control, ***P<0.001 compared with Control, ^#^*P*<0.05 compared with Ang II, ^##^*P*<0.01 compared with Ang II,^###^*P*<0.001 compared with Ang II; *n*=3.

### Caspase-1 inhibitor attenuates Ang II-induced hypertrophy in cardiomyocytes

We further investigated the involvement of pyroptosis in Ang II-induced cardiomyocyte hypertrophy. Immunofluorescence staining showed that after treatment with caspase-1 inhibitor AC-YVAD-CMK, the surface areas of cardiomyocytes were significantly decreased compared with Ang II-treated group (Figure 4A,B). The mRNA expression levels of hypertrophy related markers, including atrial natriuretic peptide (ANP), brain natriuretic peptide (BNP), and β-myosin heavy chain (β-MHC) were also down-regulated after caspase-1 inhibitor AC-YVAD-CMK treatment in cardiomyocytes (Figure 4C–E).

**Figure 4:** Caspase-1 inhibitor attenuates Ang II-induced hypertrophy in cardiomyocytes (**A**) Representative images of α-actinin and Hoechst staining in cardiomyocytes. (**B**) The statistical results of cardiomyocytes surface area in each group. (**C**) *ANP* mRNA expression in cardiomyocytes. (**D**) *BNP* mRNA expression in cardiomyocytes. (**E**) *β-MHC* mRNA expression in cardiomyocytes. GAPDH served as the internal control. **P<0.01 compared with Control, ***P<0.001 compared with Control, ^#^*P*<0.05 compared with Ang II, ^##^*P*<0.01 compared with Ang II, ^###^*P*<0.001 compared with Ang II; for (B), *n*=100 from nine separated fields; for (C–E), *n*=3.

## Discussion

Cardiac hypertrophy is an independent risk factor for cardiovascular events [18]. Therefore, exploring the molecular mechanisms of cardiac hypertrophy are vitally important. Pyroptosis is a caspase-1-dependent pro-inflammatory programmed cell death. Different from other programmed cell deaths, pyroptosis undergoes membrane blebbing and produces pyroptotic bodies prior to plasma membrane rupture [7]. Several studies demonstrated that pyroptosis plays roles in several types of diseases [16,19,20].

Caspase-1 plays an important role in regulation of cardiomyocyte biology. It was activated in hyperglycemia and doxorubicin-induced cardiac injury [16,21]. It also mediates cardiomyocyte apoptosis contributing to the progression of heart failure [22]. In addition, plenty of studies evidenced the important role and therapeutic potential of its downstream factor IL-1β in cardiac hypertrophy [23,24]. However, little was known about the role of caspase-1-induced pyroptosis in cardiac hypertrophy.

The aim of the present work was to investigate the effect of cleaved caspase-1-mediated pyroptosis in cardiac hypertrophy. TAC was used to establish a mice model of cardiac hypertrophy and cleaved caspase-1 and IL-1β expression levels were detected. The result showed that cleaved caspase-1 and IL-1β expression levels were significantly up-regulated in hypertrophic myocardium from mice. Similar results were obtained *in vitro*. Subsequently, we observed the effect of caspase-1 inhibitor on cardiac hypertrophy. Co-administration of caspase-1 inhibitor AC-YVAD-CMK could attenuate the pro-hypertrophic effect of Ang II and inhibit the abnormal expression of cleaved caspase-1 and IL-1β. These findings suggest that cleaved caspase-1-mediated pyroptosis participates in cardiac hypertrophy. Therefore, inhibition of caspase-1 may be a new strategy for prevention and treatment of cardiac hypertrophy.

Even though plenty of therapeutic targets have been identified, few of them were developed as a drug. The development of caspase-1 inhibitor was largely attributed to the researches in epilepsy and HIV infection [25,26]. VX-765 is an orally active caspase-1 inhibitor, which is well-tolerated in a 6 weeks long-phase II trial in patients with epilepsy. It may be a promising candidate for treatment of cardiac hypertrophy through the inhibition of caspase-1 and IL-1β.

In conclusion, our results provide a novel evidence that caspase-1-mediated pyroptosis plays an important role in cardiac hypertrophy, and the inhibition of caspase-1 will offer a therapeutic potential against cardiac hypertrophy.

## Abbreviations

Ang II: angiotensin II
DMEM: Dulbecco’s modified Eagle’s medium
HE: hematoxylin and eosin
HRP: horseradish peroxidase
IL-1β: interleukin-1β
TAC: transverse aortic constriction
